This article has been retracted.

# Prognostic Role of Secretory Clusterin in Multiple Human Malignant Neoplasms: A Meta-Analysis of 26 Immunohistochemistry Studies

**DOI:** 10.1371/journal.pone.0161150

**Published:** 2016-08-17

**Authors:** Jianzhong Zhang, Chenkui Miao, Aiming Xu, Kai Zhao, Zhiqiang Qin, Xiao Li, Chao Liang, Yibo Hua, Wei Chen, Chao Zhang, Yiyang Liu, Shifeng Su, Zengjun Wang, Bianjiang Liu

**Affiliations:** State Key Laboratory of Reproductive Medicine and Department of Urology, The First Affiliated Hospital of Nanjing Medical University, Nanjing. 210029, China; Universidade de Sao Paulo, BRAZIL

## Abstract

Secretory clusterin (sCLU) is a potential prognostic tumour biomarker, but results of different sCLU studies are inconsistent. We conducted this meta-analysis to evaluate the precise predictive value of sCLU. Qualified studies were identified by performing online searches in PubMed, EMBASE, and Web of Science. The selected articles were divided into three groups based on scoring method for clusterin detection. Pooled hazard ratios (HRs) with 95% confidence interval (CI) for patient survival and disease recurrence were calculated to determine the correlation between sCLU expression and cancer prognosis. Heterogeneity was assessed using *I*^*2*^ statistics, and specific heterogeneity in different groups was analysed. Elevated sCLU was significantly associated with recurrence-free survival in groups 1 and 3 (group 1: pooled HR = 1.35, 95% CI = 1.01 to 1.79; group 3: pooled HR = 1.80, 95% CI = 1.22 to 2.65). However, clusterin expression was not associated with overall survival in all three groups. Results showed that only the heterogeneity of group 2 was very strong (p = 0.013, *I*^*2*^ = 76.3%), in which the specimens were scored through sCLU staining intensity only. sCLU is a potential biomarker for tumour prognosis, and IHC methods can be more standardised if both intensity and staining proportion are considered.

## Introduction

Clusterin, coded by a highly conserved gene, was first identified in ram’s rete testis fluid[1]. Now, clusterin is widely found in various tissues and organs and is involved in a number of biological processes, including fluid transport, cell apoptosis, cell adhesion, etc[2–5]. The abnormal expression of clusterin protein is reportedly associated with Alzheimer’s disease, aging, cardiovascular diseases, inflammatory diseases, and tumourigenesis[6–10]. Clusterin protein has several isoforms arising from alternative protein splicing. Two isoforms of clusterin with opposing actions on cell apoptosis have been identified; one is secretory clusterin (sCLU), which prevents cell apoptosis, and the other is nuclear clusterin (nCLU), which induces cell apoptosis[4]. sCLU, the main isoform, has been extensively researched in the field of tumour diagnosis and prognosis considering its antiapoptotic function.

In most clinical studies, sCLU has been revealed to be a poor prognosis indicator associated with tumour relapse and metastases, including bladder cancer, prostate cancer, and lung cancer[11–18]. For instance, Matsuwaki et al. found that higher sCLU expression in the lymph-node tumour of nonsmall-cell lung cancer (NSCLC) patients predicted a higher recurrence-free survival (RFS), which suggests that sCLU is associated with enhanced NSCLC cell survival and proliferation and thus leads to poor prognosis[17]. However, some studies have presented contradictory or insignificant results, even in the same kind of malignancy. Albert et al. and Panico et al. studied NSCLC patients and found that higher sCLU expression in the original tissue specimen is associated with lower RFS. Li et al. found no significant relationship between sCLU expression and RFS[19–21]. In addition, the relationship between sCLU and overall survival (OS) has also been widely researched in various tumour studies[19–36], whose results also present contradictory results about the prognostic function of sCLU.

The role of CLU is controversial and has been previously stated and described in many reviews. Many studies have elucidated the antiapoptotic function of the sCLU and the positive association between sCLU and epithelial–mesenchymal transition (EMT), which suggest that sCLU protein can be a promoter of tumour-cell survival[37]. However, according to existing clinical data, whether sCLU acts as a good or bad indicator in clinical tumour progression is unclear. Thus, we conducted this meta-analysis to identify the specific clinical prognostic role of sCLU protein using pooled survival data. In addition, given that the method for detecting sCLU expression differs in each study especially in immunohistochemistry (IHC), we discussed the pooled data in different groups using various scoring methods and then valued the heterogeneity in each group. This technique may partly reflect the quality of a series of IHC studies using the same scoring method considering the subjectivity of IHC studies. If high heterogeneity exists or the IHC scoring results significantly differed from one another in a series of studies using the same scoring method, the group of studies can be considered hardly reproducible and subjective after excluding other factors (pathology type, an individual heterogeneous study, etc.). Subsequently, an incorrect clinical consequence ensued. The heterogeneity in each group was discussed in this meta-analysis. This is the first meta-analysis to evaluate the relationship between sCLU IHC expression and the prognosis of patients with various cancers.

## Materials and Methods

### Search strategy

This study aimed to clarify the comprehensive predictive value of sCLU or cytoplasmic clusterin in human malignant neoplasms. Online databases including PubMed, EMBASE and Web of Science were searched to identify relevant literature published until 3 April 2016. The searched keywords were “clusterin protein and (cancer or carcinoma or tumour or neoplasm) and (survival or prognosis or relapse or recurrence).” The title and abstract of the citations were inspected to identify the articles appearing to report the study of sCLU’s relationship with survival or recurrence. After a preliminary evaluation of the published papers, we found the clusterin expression was measured in various ways, including by IHC, enzyme-linked immunosorbent assay (ELISA), real-time polymerase chain reaction (qPCR), and northern blot, among which IHC is the most common method for clusterin-expression detection in the field of prognosis analyses. In this meta-analysis, we focused on papers in which IHC method was utilised for clusterin detection because of the extremely limited amount of papers in which other methods were applied. ELISA, Northern blot, and qPCR were applied in only three, three, and one paper, respectively (Fig 1). In addition, we searched literature published in Chinese to better understand the predictive role of sCLU. One study published in Chinese was finally included[22].

**Fig 1:** Flow diagram of the study selection process.

### Quality assessment

This meta-analysis was strictly performed according to the preferred reporting items of the systematic reviews and meta-analysis (PRISMA) statement. Our inclusion criteria was derived from the published guidelines (REMARK) for reporting IHC-based tumour marker studies, which was from a previously described protocol[38]. The criteria has been applied to the quality assessment of IHC-based meta-analysis in several studies before[39, 40]. The inclusion criteria were as follows: (1) a well-defined population and study design, i.e., all patients included in the study suffered a definite carcinoma and received the same therapeutic schedule, such as the same chemotherapy regimen; (2) a clear description of the IHC method, including the tissue specimens’ preparation and storage, the details of the primary antibody (specific to sCLU) and secondary antibody used, and the positive or negative control or the pictures of the staining; (3) a clear description of the scoring method of the IHC and an explicit cutoff point that differs between the positive- and negative-expression group; (4) a precise definition of the clinical endpoints examined and reporting of the resulting hazard ratio (HRs) or risk ratio values, including 95% confidence intervals (CIs) or survival curve; and (5) no overlapping with other datasets in the present study. Studies were deemed eligible according to the aforementioned criteria to maintain the quality of the meta-analysis. Given that the clusterin IHC scoring method varied among different studies, we divided the included papers in this meta-analysis into three groups according to the scoring and reporting protocols: group 1 was scored by both intensity staining and proportion of the staining cells, group 2 was scored by the staining intensity, and group 3 was scored by the proportion of staining cells.

We separately discussed the pooled data, and a sensitivity analysis for each group was conducted to prevent a highly heterogeneous study (Fig 2). In addition, we analysed the heterogeneity of each group individually by comparing their *I*^*2*^ values.

**Fig 2:** Sensitivity of each included study in three different groups. (A) Sensitivity analysis of OS in group 1. (B) Sensitivity analysis of RFS in group 1. (C) Sensitivity analysis of OS in group 2. (D) Sensitivity analysis of RFS in group3.

### Data extraction

Data were extracted from the different groups, and the extracted-data elements included the following: (1) first author’s name and publication year; (2) study population, ethnicity, nationality, disease type, and main type of pathology; (3) median or mean age of patients; (4) IHC scoring methods, cutoff definition, and follow-up time; and (5) HRs associated with upregulated clusterin expression for OS, RFS, and disease-free survival (DFS) along with their 95% CIs. In some papers that provided only Kaplan–Meier curves, the HRs and their 95% CIs were calculated using graphical survival plots as previously described[41, 42]. All these data are listed in Table 1.

**Table 1:** Main characteristics of studies included and HRs for patient OS or DFS/RFS in association with clusterin expression.

		Case number		OS		DFS/RFS					
Groups	First author, published year	High expression	Low expression	HR (95%CI)	P value	HR (95%CI)	P value	Source of HR	Disease type	Pathology type	Ethnicity
group1	Luo, 2005	32	37	2.49(0.82 to 7.55)	0.01			SC	Bladder Cancer	TCC	Asian
	Yang,2009	40	46	1.38(0.61 to 3.13)	0.03			SC	Ovarian Cancer	AdenoCA	Asian
	MIYAKE,2006	59	113	1.68(0.8 to 3.52)	0.17			SC	PCA	AdenoCA	Asian
	Zhang,2006	96	62	1.21(0.17 to 8.47)	0.00			SC	Breast Cancer	AdenoCA	Asian
	Watari,2008	21	31	1.85(0.27 to 12.94)	0.01			SC	Cervical Cancer	SqCa	Asian
	BI, 2010	47	118	1.01(0.6 to 1.71)	0.96			Reported	Gastric Cancer	AdenoCA	Asian
	He,2009	47	63	1.1(0.62 to 1.97)	0.15	1.27(0.75 to 2.15)	0.09	SC	Esophageal Cancer	SqCa	Asian
	Panico,2013	34	49	0.41(0.17 to 1.01)	0.05	0.46(0.21 to 1.00)	0.05	Reported	NSCLC	AdenoCA	Caucasian
	MIYAKE,2005	33	43			1.67(0.26 to 2.63)	0.02	Reported	PCA	AdenoCA	Asian
	Kurahashi,2005	61	70			1.65(0.68 to 4.01)	0.00	SC	Renal Cancer	RCC	Asian
	YOM,2009	97	89			1.39(0.35 to 5.59)	0.04	SC	Breast Cancer	AdenoCA	Asian
	Harada,2012	43	79			2.51(1.21 to 5.22)	0.00	SC	RCC	AdenoCA	Asian
	Matsuwaki,2014	24	40			1.55(0.74 to 2.58)	0.04	Reported	NSCLC	SqCa	Asian
group2	Albert,2007	44	62	0.487(0.27 to 0.89)	0.01	0.354(0.12 to 1.2)	0.02	Reported	NSCLC	SqCa	Caucasian
	Partheen, 2008	NM	NM	0.29(0.08 to 1.08)	0.00			SC	Ovarian Cancer	AdenoCA	Caucasian
	Kevans,2009	136	115	2.88(1.48 to 5.61)	0.00			SC	Colorectal Cancer	AdenoCA	Caucasian
	Watari,2010	14	32	2.79(0.4 to 19.19)	0.01			SC	Cervical Cancer	SqCa	Asian
	Hassan,2011	15	32	2.22(0.12 to 42.52)	0.04			SC	Ovarian Cancer	AdenoCA	Asian
	Jin,2012	17	35	0.65(0.283 to 1.49)	0.31			Reported	Pancreatic Cancer	AdenoCA	Asian
	Watari,2012	8	26	3.32(0.95 to 11.69)	0.02			SC	Cervical Cancer	SqCa	Asian
	Tobisawa,2013	92	13	4.1(1.27 to 13.27)	0.02			Reported	T-cell lymphoma	MF	Asian
group3	Xie,2001	16	17	0.37(0.11 to 1.32)	0.01			SC	Pancreatic Cancer	AdenoCA	Asian
	KRÜGER,2006	29	89			2.69(0.97 to 7.51)	0.05	Reported	Bladder Cancer	TCC	Caucasian
	KRÜGER,2006	36	105			2.19(1.05 to 4.57)	0.06	SC	Breast Cancer	AdenoCA	Caucasian
	Redondo,2009	31	72			2.01(1.03 to 3.9)	0.04	Reported	Colorectal Cancer	AdenoCA	Caucasian
	Li,2010	70	51	1.63(0.22 to 12.03)	0.37	0.92(0.41 to 2.09)	0.62	SC	NSCLC	AdenoCA	Asian

AdenoCA, adenocarcinoma; DFS, disease-free survival; HR (high vs low); NM, not mentioned; NSCLC, non-small cell lung cancer; OS, overall survival; PCA, prostate carcinoma; RCC, renal cell carcinoma; RFS, relapse-free survival; SC, survival curve; SqCa, squamous carcinoma.

### Statistical analysis

Fixed-effect summary HRs and 95% CIs were calculated using the Mantel–Haenszel method and the random-effect model based on the DerSimonian–Laird method according to heterogeneity among the pooled studies[43]. Heterogeneity was assessed using Higgins I^2^ statistic and Cochran Q test[44]. A random-effect model was applied if significant heterogeneity was observed (p<0.10 or *I*^*2*^ >50%); otherwise, the fixed-effect model was utilised. An HR value greater than 1 indicated poor outcome for the upregulated to the downregulated clusterin expression and was considered statistically significant if the 95% CI did not include 1, with P < 0.05. Egger’s linear regression test was applied to estimate the publication bias with a funnel plot[45]. A p value less than 0.05 was considered statistically significant. The meta-analyses were carried out with Stata12 (StataCorp LP, College Station, TX, USA).

## Result

### Summary of the enrolled studies

Our search of clusterin prognostic literature yielded 454 manuscripts (S1 File) using PubMed, EMbase, and Web of Science. Sixty articles were identified through primary title and abstract evaluation, and studies were excluded if they were review articles, did not use a human subject, or were not related to the current meta-analysis. After a primary evaluation, full text articles were obtained for these 60 manuscripts; 11 studies were excluded secondarily because they did not provide the survival data (HRs and survival curves), 12 studies were excluded because they were not directly related to the specific outcome, and 13 articles were excluded because they did not use the IHC method for sCLU detection. Ultimately, all remaining articles were checked secondarily, and no overlapping datasets were found (Fig 1). A total of 26 articles were included in our meta-analysis finally.

The main features of the 26 enrolled articles are systematically summarised in Table 1. Eight studies focused on RFS, fourteen reported patient OS, and four investigated OS and DFS. Among these studies, a total of 2631 participants were included; 19 studies focused on Asians, and 7 evaluated Caucasians. The malignant neoplasms assessed in these studies included bladder cancer, ovarian cancer, prostate cancer, breast cancer, cervical cancer, gastric cancer, esophageal cancer, colorectal cancer, lymphoma, and NSCLC. Sixteen articles focused on the pathological type of adenocarcinoma (adenoCA), six assessed squamous carcinoma (SqCa), two evaluated transitional cell carcinoma (TCC), one focused on lymphoma and one detected renal cell carcinoma(RCC). Three groups were divided as previously described in this analysis according to the IHC scoring method. In total group 1 had 13 studies, group 2 had 8 studies, and group 3 had 5 studies.

### Sensitivity analyses

Our sensitivity analyses in the three different groups (both in OS and DFS/RFS analyses) did not indicate alterations in the results if any individual study was excluded (Fig 2), suggesting that no single study significantly influenced the pooled HR or the 95% CI.

### Recurrence associated with sCLU expression

A total of 11 studies were included in the DFS/RFS analysis. Both groups 1 and 3 revealed a risk factor of increased sCLU expression (group 1: pooled HR = 1.35, 95% CI = 1.01 to 1.79; group 3: pooled HR = 1.80, 95% CI = 1.22 to 2.65), as determined by a fixed-effect model (group 1: p = 0.100, *I*^*2*^ = 43.6%; Group 3: p = 0.311, *I*^*2*^ = 16.2%) (Fig 3) in a combined analysis. Group 2 involved only one study (HR = 0.354, 95% CI = 0.12 to 1.2).

**Fig 3:** Forest plots of merged analyses of disease-free survival (DFS)/relapse-free survival (RFS) in association with sCLU expression in different groups. Forest plots of merged analyses of overall survival (OS). Squares and horizontal lines represent study-specific HRs and 95% CIs, respectively. The areas of the squares correspond to weights, and the diamonds represent overall HRs and 95% CIs. (A) Forest plots of merged analyses of RFS/DFS in group 1. (B) Forest plots of merged analyses of RFS/DFS in group3.

### OS associated with sCLU expression

A total of 19 studies were included in the OS analysis. In all groups, no significant relationship existed between sCLU and OS (group 1: pooled HR = 1.13, 95% CI = 0.86 to 1.50; group 2: pooled HR = 1.14, 95% CI = 0.82 to 1.60; group 3: pooled HR = 1.64, 95% CI = 0.95 to 2.83), as determined by a fixed-effect model in groups1 and 3 (p = 0.276, *I*^*2*^ = 19.4%; group 3: p = 0.217, *I*^*2*^ = 34.3%) and a random-effect model in groups 2 (p = 0.000, *I*^*2*^ = 76.3%) (Fig 4). Considering the high heterogeneity of group 2, a stratified analysis was conducted in group2 through ethnicity and pathology disease, and *I*^*2*^ was still high in each subgroup (Fig 5), which made the subgroups’ HRs difficult to pool.

**Fig 4:** Forest plots of merged analyses of overall survival (OS) in association with sCLU expression in different groups. Forest plots of merged analyses of disease-free survival (DFS)/relapse-free survival (RFS). Squares and horizontal lines represent study-specific HRs and 95% CIs, respectively. The areas of the squares correspond to weights, and the diamonds represent overall HRs and 95% CIs. (A) Forest plots of merged analyses of overall survival (OS) in group 1. (B) Forest plots of merged analyses of overall survival (OS) in group 2. (C) Forest plots of merged analyses of overall survival (OS) in group3.

**Fig 5:** Subgroup analyses of group 2. (A) shows the pathology-type subgroup analysis, and (B) shows the ethnicity subgroup analysis.

### Publication bias

The funnel plots of the publication bias are presented in Fig 6 respectively. They showed no obvious publication bias.

**Fig 6:** Begg’s funnel plots of the publication bias. Begg’s funnel plots of the publication bias for overall merged analysis of OS or DFS/RFS. Each point represents a separate study. About the OS analysis, (A) and (B) represents group 1 and group 2 respectively. About the DFS/RFS analysis, (C) and (D) represents group 1 and group 3 respectively.

## Discussion

Tumour relapse and metastases always suggest a bad outcome for patients suffering from malignancy. Discovering an effective biomarker that can predict tumour progression is important so that an appropriate treatment can be applied. Patients with higher-risk biomarker expression can receive a more extensive treatment and be required of more frequent follow-up visits. The role of CLU in tumour prognosis is controversial and has been previously stated in many reviews. On one side, many studies have demonstrated that sCLU promoted tumourigenesis. For instance, sCLU has been found abnormally upregulated in various advance-stage and metastatic cancers and proven to be a biomarker for tumourigenesis and progression over the past decades[46]. The association of sCLU expression with tumour prognosis may be partially due to its biological function, especially in the field of antiapoptosis. sCLU protects tumour cells from apoptosis by stablising Ku70/Bax to prevent its actions on the mitochondrial membrane activating the phosphatidylinositol 3-kinase/protein kinase B pathway, modulating extracellular signal-regulated kinase 1/2 signaling and matrix metallopeptidase-9 expression, and increasing angiogenesis[4]. On the other side, though sCLU was found up-regulated in various advance-stage and metastatic cancers in many studies[46], data available on the Oncomine database showed that CLU transcripts were down-regulated in tumours as compared to normal tissues in many microarray analyses (www.oncomine.org). According to existing clinical data, whether sCLU acts as a good or bad indicator in clinical tumour progression is still controversial.

Recently, many studies have facilitated advance in the research of CLU. First, several CLU mRNA isoforms have been identified, including Isoform 1, Isoform 2, and Isoform 11036[47]. Subsequently studies have been performed measuring the amount of different mRNAs coding for CLU, showing huge differences in mRNA isoform expression in different experimental systems[48, 49]. Second, specific mRNA CLU isoforms are also differentially regulated in cancer cells. At least two putative promoter regions have been discovered, respectively surrounding the transcription start site of Isoform 1 and Isoform 2[48]. In addition, CLU production process is dynamic and complicated and any factors related to sCLU production or excretion can influence sCLU expression[50]. Moreover, the regulation of NF-kB-activation is another proposed function of CLU. However, both NF-kB-stimulatory and -inhibitory properties have been described, which might be aroused from different CLU isoforms[51, 52]. All the aforementioned data showed that the mechanism of CLU in tumour is complicated and challenging.

Meta-analysis, as an effective tool, can provide more dependable results than a single research especially in explaining controversial conclusions. As a consequence, we took advantage of meta-analysis to analyse the possible association between sCLU and tumour prognosis. In the present work, actual clinical data showed contradictory results (Table 1). This is the first meta-analysis to evaluate the relationship between sCLU IHC expression and the prognosis of patients with various cancers. Our RFS/DFS analyses revealed a pooled HR of 1.58 in group 1 and 1.79 in group 3, which suggested that sCLU acted as a bad outcome indicator in tumour relapse and metastases in both groups. OS analyses in the three different groups showed contradictory results (HR = 1.13, 1.14, and 1.64 in groups 1, 2, and 3, respectively). However, the result was not significant in all three groups. Insufficiently strong HRs and the accompanying insignificant CIs may imply that the role of sCLU in human malignancies is complex and controversial. sCLU can be a prognostic biomarker for relapse and metastasis, but its action on patient survival was weak based on our analysis.

We further analysed the heterogeneity of the three groups in the OS-related studies. Results showed that the heterogeneity of group 2 and group 3 were very strong (p = 0.000, *I*^*2*^ = 76.3%), in which the specimens were scored through sCLU staining intensity only. Secondary analyses were conducted to identify the origin of the heterogeneity. Subgroup analyses showed that the ethnicity and pathology subgroups did not obtain a smaller *I*^*2*^ (Fig 5). Meanwhile, sensitivity analysis results showed that no single heterogeneous study existed. This finding might suggest that the scoring method that only used staining intensity as an index can be inappropriate. By contrast contrary, scoring method both using staining proportion and intensity as a standard of the specimen can be more objective and accurate.

To distinguish the positive or negative expression of sCLU protein, these IHC studies in group 2 set a cutoff point according to expression intensity. The specific intensity of each tissue specimen was described as negative, weak, moderate, or strong according to a positive or negative control. Among them, negative- or weak-expression specimens were incorporated into the negative-expression group, and the others were incorporated into the positive group. Given that specific staining intensity was identified subjectively, the result changed from different pathologists and thus increased the heterogeneity of the studies in group 2.

By contrast, the studies in groups 1 and 3 used staining-cell proportion as a scoring method or as part of the scoring method, which was relatively objective. In group 3, the proportion of staining cells was recorded, and if >10% cells were stained, the specimen was included in the positive group. In group 1, both intensity and proportion of staining cells were considered. Usually, intensity and proportion were scored separately in each specimen, and then the score values were added or multiplied. A median or mean value was then set as a cutoff point in these situations.

Finally, our conclusions should be considered with caution because of the following limitations. First, the IHC scoring methods and the cutoff points differed among various studies, and these factors caused by IHC substantially increased heterogeneity in our analyses. Although we divided our enrolled studies into three groups from the IHC methods, heterogeneity cannot be completely avoided because each study had little differences in scoring method. For instance, in group 1, some researchers used three as a cutoff point, whereas some chose the median score. Second, IHC intensity was judged by a pathologist, which inevitably made the IHC results subjective. Third, the number of enrolled participants was smaller in each group. Heterogeneity also arose from the pathological type and ethnicity.

## Conclusions

Our results suggested that sCLU was a potential biomarker for malignancy RFS/DFS. IHC methods can also become more standardised if both intensity and the proportion can be considered.

## Supporting Information

S1 File Titles of the potential relevant articles. (DOC)

## References

[1] FritzIB, BurdzyK, SetchellB, BlaschukO. Ram rete testis fluid contains a protein (clusterin) which influences cell-cell interactions in vitro. Biology of reproduction. 1983;28(5):1173–88. .687131310.1095/biolreprod28.5.1173

[2] TrougakosIP, GonosES. Clusterin/apolipoprotein J in human aging and cancer. The international journal of biochemistry & cell biology. 2002;34(11):1430–48. .1220003710.1016/s1357-2725(02)00041-9

[3] SalaA, BettuzziS, PucciS, ChaykaO, DewsM, Thomas-TikhonenkoA. Regulation of CLU gene expression by oncogenes and epigenetic factors implications for tumorigenesis. Advances in cancer research. 2009;105:115–32. 10.1016/S0065-230X(09)05007-6 19879426PMC3426299

[4] KoltaiT. Clusterin: a key player in cancer chemoresistance and its inhibition. OncoTargets and therapy. 2014;7:447–56. 10.2147/OTT.S58622 24672247PMC3964162

[5] de SilvaHV, HarmonyJA, StuartWD, GilCM, RobbinsJ. Apolipoprotein J: structure and tissue distribution. Biochemistry. 1990;29(22):5380–9. .197445910.1021/bi00474a025

[6] BagyinszkyE, YounYC, AnSS, KimS. The genetics of Alzheimer's disease. Clinical interventions in aging. 2014;9:535–51. 10.2147/CIA.S51571 24729694PMC3979693

[7] LiX, MaY, WeiX, LiY, WuH, ZhuangJ, et al Clusterin in Alzheimer's disease: a player in the biological behavior of amyloid-beta. Neuroscience bulletin. 2014;30(1):162–8. 10.1007/s12264-013-1391-2 .24353014PMC5562576

[8] ParkS, MathisKW, LeeIK. The physiological roles of apolipoprotein J/clusterin in metabolic and cardiovascular diseases. Reviews in endocrine & metabolic disorders. 2014;15(1):45–53. 10.1007/s11154-013-9275-3 .24097125

[9] TrougakosIP, GonosES. Regulation of clusterin/apolipoprotein J, a functional homologue to the small heat shock proteins, by oxidative stress in ageing and age-related diseases. Free radical research. 2006;40(12):1324–34. 10.1080/10715760600902310 .17090421

[10] LinCC, TsaiP, SunHY, HsuMC, LeeJC, WuIC, et al Apolipoprotein J, a glucose-upregulated molecular chaperone, stabilizes core and NS5A to promote infectious hepatitis C virus virion production. Journal of hepatology. 2014;61(5):984–93. 10.1016/j.jhep.2014.06.026 .24996046

[11] KrugerS, MahnkenA, KauschI, FellerAC. Value of clusterin immunoreactivity as a predictive factor in muscle-invasive urothelial bladder carcinoma. Urology. 2006;67(1):105–9. 10.1016/j.urology.2005.04.043 .16413343

[12] KrugerS, OlaV, FischerD, FellerAC, FriedrichM. Prognostic significance of clusterin immunoreactivity in breast cancer. Neoplasma. 2007;54(1):46–50. .17203891

[13] RedondoM, RodrigoI, AlcaideJ, TellezT, RoldanMJ, FunezR, et al Clusterin expression is associated with decreased disease-free survival of patients with colorectal carcinomas. Histopathology. 2010;56(7):932–6. 10.1111/j.1365-2559.2010.03565.x .20497247

[14] MiyakeH, YamanakaK, MuramakiM, KurahashiT, GleaveM, HaraI. Enhanced expression of the secreted form of clusterin following neoadjuvant hormonal therapy as a prognostic predictor in patients undergoing radical prostatectomy for prostate cancer. Oncology reports. 2005;14(5):1371–5. .16211311

[15] YomCK, WooHY, MinSY, KangSY, KimHS. Clusterin overexpression and relapse-free survival in breast cancer. Anticancer research. 2009;29(10):3909–12. .19846927

[16] HaradaK, MiyakeH, KusudaY, FujisawaM. Expression of epithelial-mesenchymal transition markers in renal cell carcinoma: impact on prognostic outcomes in patients undergoing radical nephrectomy. BJU international. 2012;110(11 Pt C):E1131–7. 10.1111/j.1464-410X.2012.11297.x .22712620

[17] MatsuwakiR, IshiiG, ZenkeY, NeriS, AokageK, HishidaT, et al Immunophenotypic features of metastatic lymph node tumors to predict recurrence in N2 lung squamous cell carcinoma. Cancer science. 2014;105(7):905–11. 10.1111/cas.12434 24814677PMC4317916

[18] KurahashiT, MuramakiM, YamanakaK, HaraI, MiyakeH. Expression of the secreted form of clusterin protein in renal cell carcinoma as a predictor of disease extension. BJU international. 2005;96(6):895–9. Epub 2005/09/13. 10.1111/j.1464-410X.2005.05733.x .16153225

[19] AlbertJM, GonzalezA, MassionPP, ChenH, OlsonSJ, ShyrY, et al Cytoplasmic clusterin expression is associated with longer survival in patients with resected non small cell lung cancer. Cancer epidemiology, biomarkers & prevention: a publication of the American Association for Cancer Research, cosponsored by the American Society of Preventive Oncology. 2007;16(9):1845–51. 10.1158/1055-9965.EPI-07-0146 .17855704

[20] LiH, LiuS, ZhuX, YangS, XiangJ, ChenH. Clusterin immunoexpression and its clinical significance in patients with non-small cell lung cancer. Lung. 2010;188(5):423–31. 10.1007/s00408-010-9248-1 .20614220

[21] PanicoF, CasaliC, RossiG, RizziF, MorandiU, BettuzziS, et al Prognostic role of clusterin in resected adenocarcinomas of the lung. Lung Cancer. 2013;79(3):294–9. Epub 2013/01/02. 10.1016/j.lungcan.2012.11.024 .23276503

[22] LuoJH, XieD, ChenW, DaiYP, LiXF, TaoY, et al [Correlation of clusterin expression to prognosis of bladder carcinoma]. Ai zheng = Aizheng = Chinese journal of cancer. 2005;24(6):743–7. Epub 2005/06/11. .15946493

[23] YangGF, LiXM, XieD. Overexpression of clusterin in ovarian cancer is correlated with impaired survival. International journal of gynecological cancer: official journal of the International Gynecological Cancer Society. 2009;19(8):1342–6. 10.1111/IGC.0b013e3181a83ed9 .20009887

[24] MiyakeH, MuramakiM, KurahashiT, YamanakaK, HaraI, GleaveM, et al Expression of clusterin in prostate cancer correlates with Gleason score but not with prognosis in patients undergoing radical prostatectomy without neoadjuvant hormonal therapy. Urology. 2006;68(3):609–14. 10.1016/j.urology.2006.03.017 .16979705

[25] ZhangS, ZhangD, ZhuY, GuoH, ZhaoX, SunB. Clusterin expression and univariate analysis of overall survival in human breast cancer. Technology in cancer research & treatment. 2006;5(6):573–8. .1712143310.1177/153303460600500604

[26] WatariH, OhtaY, HassanMK, XiongY, TanakaS, SakuragiN. Clusterin expression predicts survival of invasive cervical cancer patients treated with radical hysterectomy and systematic lymphadenectomy. Gynecologic oncology. 2008;108(3):527–32. 10.1016/j.ygyno.2007.11.026 .18177691

[27] BiJ, GuoAL, LaiYR, LiB, ZhongJM, WuHQ, et al Overexpression of clusterin correlates with tumor progression, metastasis in gastric cancer: a study on tissue microarrays. Neoplasma. 2010;57(3):191–7. .2035326810.4149/neo_2010_03_191

[28] HeLR, LiuMZ, LiBK, RaoHL, LiaoYJ, ZhangLJ, et al Clusterin as a predictor for chemoradiotherapy sensitivity and patient survival in esophageal squamous cell carcinoma. Cancer science. 2009;100(12):2354–60. 10.1111/j.1349-7006.2009.01349.x .19793084PMC11158670

[29] PartheenK, LevanK, OsterbergL, ClaessonI, FalleniusG, SundfeldtK, et al Four potential biomarkers as prognostic factors in stage III serous ovarian adenocarcinomas. International journal of cancer Journal international du cancer. 2008;123(9):2130–7. 10.1002/ijc.23758 .18709641

[30] WatariH, KanumaT, OhtaY, HassanMK, MitamuraT, HosakaM, et al Clusterin expression inversely correlates with chemosensitivity and predicts poor survival in patients with locally advanced cervical cancer treated with cisplatin-based neoadjuvant chemotherapy and radical hysterectomy. Pathology oncology research: POR. 2010;16(3):345–52. 10.1007/s12253-009-9235-0 .20058210

[31] HassanMK, WatariH, HanY, MitamuraT, HosakaM, WangL, et al Clusterin is a potential molecular predictor for ovarian cancer patient's survival: targeting clusterin improves response to paclitaxel. Journal of experimental & clinical cancer research: CR. 2011;30:113 10.1186/1756-9966-30-113 22185350PMC3287343

[32] JinJ, KimJM, HurYS, ChoWP, LeeKY, AhnSI, et al Clinical significance of clusterin expression in pancreatic adenocarcinoma. World journal of surgical oncology. 2012;10:146 10.1186/1477-7819-10-146 22799602PMC3436747

[33] WatariH, KinoshitaR, HanY, WangL, HosakaM, TaguchiH, et al Prognostic significance of clusterin expression in advanced-stage cervical cancer treated with curative intended radiotherapy. International journal of gynecological cancer: official journal of the International Gynecological Cancer Society. 2012;22(3):465–70. 10.1097/IGC.0b013e31821a03d9 .21633299

[34] TobisawaS, HonmaM, Ishida-YamamotoA, SaijoY, IizukaH. Prognostic factors in 105 Japanese cases of mycosis fungoides and Sezary syndrome: clusterin expression as a novel prognostic factor. Journal of dermatological science. 2013;71(3):160–6. 10.1016/j.jdermsci.2013.04.020 .23702390

[35] XieMJ, MotooY, SuSB, MouriH, OhtsuboK, MatsubaraF, et al Expression of clusterin in human pancreatic cancer. Pancreas. 2002;25(3):234–8. .1237053310.1097/00006676-200210000-00004

[36] KevansD, FoleyJ, TenniswoodM, SheahanK, HylandJ, O'DonoghueD, et al High clusterin expression correlates with a poor outcome in stage II colorectal cancers. Cancer epidemiology, biomarkers & prevention: a publication of the American Association for Cancer Research, cosponsored by the American Society of Preventive Oncology. 2009;18(2):393–9. Epub 2009/01/22. 10.1158/1055-9965.epi-08-0302 .19155441

[37] WangC, JiangK, KangX, GaoD, SunC, LiY, et al Tumor-derived secretory clusterin induces epithelial-mesenchymal transition and facilitates hepatocellular carcinoma metastasis. The international journal of biochemistry & cell biology. 2012;44(12):2308–20. 10.1016/j.biocel.2012.09.012 .23010347

[38] McShaneLM, AltmanDG, SauerbreiW, TaubeSE, GionM, ClarkGM, et al REporting recommendations for tumour MARKer prognostic studies (REMARK). British journal of cancer. 2005;93(4):387–91. 10.1038/sj.bjc.6602678 16106245PMC2361579

[39] JamiesonNB, CarterCR, McKayCJ, OienKA. Tissue biomarkers for prognosis in pancreatic ductal adenocarcinoma: a systematic review and meta-analysis. Clinical cancer research: an official journal of the American Association for Cancer Research. 2011;17(10):3316–31. 10.1158/1078-0432.CCR-10-3284 .21444679

[40] SteelsE, PaesmansM, BerghmansT, BranleF, LemaitreF, MascauxC, et al Role of p53 as a prognostic factor for survival in lung cancer: a systematic review of the literature with a meta-analysis. The European respiratory journal. 2001;18(4):705–19. .1171617710.1183/09031936.01.00062201

[41] WilliamsonPR, SmithCT, HuttonJL, MarsonAG. Aggregate data meta-analysis with time-to-event outcomes. Statistics in medicine. 2002;21(22):3337–51. 10.1002/sim.1303 .12407676

[42] TierneyJF, StewartLA, GhersiD, BurdettS, SydesMR. Practical methods for incorporating summary time-to-event data into meta-analysis. Trials. 2007;8:16 10.1186/1745-6215-8-16 17555582PMC1920534

[43] DerSimonianR, LairdN. Meta-analysis in clinical trials. Controlled clinical trials. 1986;7(3):177–88. .380283310.1016/0197-2456(86)90046-2

[44] HigginsJP, ThompsonSG, DeeksJJ, AltmanDG. Measuring inconsistency in meta-analyses. Bmj. 2003;327(7414):557–60. 10.1136/bmj.327.7414.557 12958120PMC192859

[45] EggerM, Davey SmithG, SchneiderM, MinderC. Bias in meta-analysis detected by a simple, graphical test. Bmj. 1997;315(7109):629–34. 931056310.1136/bmj.315.7109.629PMC2127453

[46] DjeuJY, WeiS. Clusterin and chemoresistance. Advances in cancer research. 2009;105:77–92. 10.1016/S0065-230X(09)05005-2 19879424PMC3889866

[47] RizziF, ColettaM, BettuzziS. Chapter 2: Clusterin (CLU): From one gene and two transcripts to many proteins. Advances in cancer research. 2009;104:9–23. Epub 2009/11/03. 10.1016/s0065-230x(09)04002-0 .19878770

[48] BonaciniM, ColettaM, RamazzinaI, NaponelliV, ModernelliA, DavalliP, et al Distinct promoters, subjected to epigenetic regulation, drive the expression of two clusterin mRNAs in prostate cancer cells. Biochimica et biophysica acta. 2015;1849(1):44–54. Epub 2014/12/03. 10.1016/j.bbagrm.2014.11.003 .25464035

[49] FuzioP, NapoliA, CiampolilloA, LattaruloS, PezzollaA, NuzzielloN, et al Clusterin transcript variants expression in thyroid tumor: a potential marker of malignancy? BMC Cancer. 2015;15:349 Epub 2015/05/03. 10.1186/s12885-015-1348-0 ; PubMed Central PMCID: PMCPmc4422431.25934174PMC4422431

[50] BettuzziS, RizziF. Chapter 5: Nuclear CLU (nCLU) and the fate of the cell. Advances in cancer research. 2009;104:59–88. Epub 2009/11/03. 10.1016/s0065-230x(09)04005-6 .19878773

[51] SantilliG, AronowBJ, SalaA. Essential requirement of apolipoprotein J (clusterin) signaling for IkappaB expression and regulation of NF-kappaB activity. The Journal of biological chemistry. 2003;278(40):38214–9. Epub 2003/07/29. 10.1074/jbc.C300252200 .12882985

[52] ZoubeidiA, EttingerS, BeraldiE, HadaschikB, ZardanA, KlompLW, et al Clusterin facilitates COMMD1 and I-kappaB degradation to enhance NF-kappaB activity in prostate cancer cells. Molecular cancer research: MCR. 2010;8(1):119–30. Epub 2010/01/14. 10.1158/1541-7786.mcr-09-0277 ; PubMed Central PMCID: PMCPmc2808437.20068069PMC2808437

